# *Apocynum* Leaf Extract Suppresses the Progress of Atherosclerosis in Rats via the FKN/SYK/p38 Signal Pathway

**DOI:** 10.1155/2021/5524226

**Published:** 2021-11-03

**Authors:** Dan Zhang, Zehui Gu, Jianxin Wang, Yang Zhang, Yang Zheng

**Affiliations:** ^1^Department of Cardiovascular, The First Hospital of Jilin University, Changchun, China; ^2^Department of Cardiovascular, Changchun Center Hospital, Changchun, China; ^3^Department of Pathology, The Third Affiliated Hospital of Jinzhou Medical University, Jinzhou, Liaoning 121000, China; ^4^Department of Pharmacy, Jilin Cancer Hospital, Changchun, Jilin 130021, China; ^5^Department of Vascular Surgery, The First Hospital of Jilin University, Changchun, China

## Abstract

To investigate the antiatherosclerotic effects of flavonoids extracted from *Apocynum venetum* (AVF) leaves in atherosclerotic rats and the underlying mechanisms, a total of 72 male Wistar rats were randomly divided into six groups: control group, model group, simvastatin group, low-dose AVF group, medium-dose AVF group, and high-dose AVF group. Atherosclerosis in rats was induced with a high-fat diet and an intraperitoneal injection of VD_3_ once daily for three contiguous days at a total injection dose of 70 U/kg. At the end of the 13^th^ week, total serum cholesterol (TC), triglyceride (TG), low-density lipoprotein cholesterol (LDL-C), and high-density lipoprotein cholesterol (HDL-C) contents were measured. The hematoxylin-eosin (HE) staining was applied to evaluate the morphological changes. The ELISA method was used to detect related inflammatory factors and oxidative stress indicators. The corresponding protein expression and the mRNA level were detected by western blot analysis and reverse transcriptase PCR. HE staining showed that the thoracic aorta wall was thickened, and the aortic subendothelial foam cells and lipid vacuoles were reduced in the medium/high-AVF groups. Similarly, the TC, TG, LDL-C, and malondialdehyde (MDA) levels in the model group were significantly higher, but the HDL-C level and superoxide dismutase (SOD) activity were lower than those of the control group, and these effects were ameliorated by treatment with simvastatin or AVF. ELISA results showed that compared with the control group, the model group C-reactive protein (CRP), interleukin-6 (IL-6), and tumor necrosis factor-*α* (TNF-*α*) results were significantly increased, and the medium AVF and high AVF could significantly reduce the expression of related inflammatory factors. The AVF inhibited intercellular cell adhesion molecule-1 (ICAM-1), vascular cell adhesion molecule-1 (VCAM-1), and E-selectin mRNA and related protein expression in the aorta in atherosclerotic rats. Western blot analysis also showed that AVF can significantly reduce the protein expression of fractalkine (FKN), spleen tyrosine kinase (SYK), and p38 mitogen-activated protein kinase (p38) in the rat aorta. We believe that the AVF can effectively reduce blood lipid levels in rats with atherosclerosis and delay atherosclerotic progression by inhibiting excessive inflammatory factors and inhibiting related adhesion factors. The underlying mechanism may be related to the FKN/SYK/p38 signaling pathway activity. Our results contribute to validating the traditional use of the *Apocynum* leaf extract in the treatment of atherosclerosis.

## 1. Introduction

Atherosclerosis (AS) is a systemic and diffuse arterial wall lesion caused by the accumulation of cholesterol in the intima of the artery and its branch vessels. It is usually accompanied by the proliferation of smooth muscle cells in the intima, subsequent thickening of the arterial vessels, and yellow AS plaques. The pathogenesis of AS is a complicated process, which is believed to be multifactorial. However, it is agreed that lipid metabolism disorders and inflammatory reactions are the pathological basis of AS [1]. In particular, the formation of foam cells, including macrophages and other cell types such as endothelial and vascular smooth muscle cells that contain deposited free and esterified cholesterol [2], plays an essential role in the development of AS [3]. Thus, efforts have been made to search for solutions to prevent lipid metabolism disorders and inflammatory reactions.

Flavonoids are polyphenolic phytochemicals extensively distributed in plants, including vegetables and fruits such as flowers, seeds, and nuts. They have been shown to exhibit a broad spectrum of biological properties. In cardiovascular research, recent studies have shown that flavonoids exhibit several physical activities, including reducing vascular fragility and abnormal permeability, dilating the coronary artery, and diminishing platelet aggregation and free radical oxidation [4–7]. For example, Wang et al. [8] found that total flavonoids of *Astragalus* ameliorate AS by reducing the area of AS plaques and decreasing the circulating levels of TG and TC.

*Apocynum venetum* L. (Luobuma and dogbane), a plant species of the Apocynaceae family, is widely distributed in China. *Apocynum venetum* (AVF) leaf extracts are used as additives in tea and for medicinal purposes. In modern medicine, AVF is used to treat hypertension, palpitations, insomnia, and neurasthenia [9–11]. Kwan et al. [12] demonstrated that the endothelium-dependent relaxation induced by AVF was potent with a maximal rate of relaxation occurring at 10 *μ*g/mL, which could be inhibited by the NO synthase inhibitor NG-nitro-L-arginine (L-NAME) and the K^+^ channel blocker tetramethylammonia. It has been proposed that this effect could be due to its nitric oxide-releasing and superoxide-scavenging properties. Therefore, in this study, we aimed to explore the impacts of AVF on AS in a rat AS model induced by vitamin D3 (VD_3_) and HCD feeding and the related mechanisms.

## 2. Materials and Methods

### 2.1. Establishment of an Atherosclerosis Model and Experimental Groups

Seventy-two SPF-grade healthy male Wistar rats weighing 180–200 g were purchased from the Experimental Animal Center of Jilin University. All animals were individually caged, had free access to drinking water, and were weighed weekly. After one week of adaptive feeding, the rats were randomly divided into the following six groups: control group (CON), model group (MOD), simvastatin group (SIM), and low-, medium-, and high-dose AVF-treated groups (low AVF, medium AVF, and high AVF) (12 rats per group). Except for the CON group, the animals received an intraperitoneal injection of VD_3_ once daily for three contiguous days at a total injection dose of 70 U/kg and were fed a high-fat diet until the end of the experiment. The 12 rats of the CON group were intraperitoneally injected with an equal volume of normal saline and fed normal feed. During the experiment, animals in the low-, medium-, and high-dose AVF groups received daily gavage of AVF at doses of 25, 50, and 100 mg/kg/d, respectively, and animals in the SIM group received simvastatin at 4 mg/kg (gavage). The dosage of AVF is mainly based on the therapeutic effect of AVF on cardiovascular diseases in previous articles. Zhang et al. studied the protection of AVF against pirarubicin-induced cardiotoxicity. The doses of AVF were 25 mg/kg, 50 mg/kg, and 100 mg/kg [7]. Kim et al. used 70 mg/kg AVF to explore its antihypertensive pharmacological effects [13]. The high-fat diet comprised 80.8% basic diet, 3.5% cholesterol, 10% lard, 0.2% propylthiouracil, 0.5% sodium cholate, and 5% white granulated sugar. The modeling method used in this experiment was redesigned by our laboratory based on the previous modeling methods and had been recognized by peers. Hu et al. used this method to replicate the rat model of atherosclerosis and verified the antiatherosclerotic effect of icariin [14]. The study was approved by the Animal Care and Ethics Committee of Jilin University (Changchun, China; Grant no. 20170503) and followed the National Institutes of Health Guidelines for the Care and Use of Laboratory Animals. All experimental animals were euthanized by inhalation of CO_2_ (30% volume displacement per minute).

### 2.2. Reagents

Total cholesterol (TC), triglyceride (TG), low-density lipoprotein cholesterol (LDL-C), high-density lipoprotein cholesterol (HDL-C), superoxide dismutase (SOD), and malonaldehyde (MDA) test kits were purchased from Nanjing Jiancheng Bioengineering Institute, China. VD_3_ injection was purchased from Shanghai General Pharmaceutical, China. Simvastatin tablets were purchased from Merck, Hangzhou, China. Sodium cholate and cholesterol were purchased from Sigma, USA. The antibody of intercellular cell adhesion molecule-1 (ICAM-1), vascular cell adhesion molecule-1 (VCAM-1), E-selectin, fractalkine (FKN), spleen tyrosine kinase (SYK), and p38 mitogen-activated protein kinase (p38) were purchased from Abcam, USA. C-reactive protein (CRP), interleukin-6 (IL-6), and tumor necrosis factor-*α* (TNF-*α*) determination kits were purchased from Shanghai Meixin Biological Engineering, China. *Apocynum venetum* flavonoids (AVF, flavonoid content ≥72%) were purchased from Nanjing Jingzhu Biotechnology Co., Ltd., China.

### 2.3. Blood Lipid Examination

When the experiment was terminated at the end of the 13^th^ week, serum was collected from each group (2000 rpm, 15 min, 4°C). Serum TC and TG, LDL-C, and HDL-C contents were measured according to the kit instructions.

### 2.4. Morphological Examination

The full length of the rat thoracic aorta is approximately 2 cm. The proximal end (0.5 cm) was fixed with 10% formalin, embedded in paraffin, and prepared as 5 *μ*m-thick sections. The sections were subjected to serial alcohol deparaffinization and stained with hematoxylin-eosin (HE). Differences in histology between the rat aortic tissues of various groups were observed under a light microscope.

### 2.5. ELISA Detection of Inflammatory Factors and Oxidative Stress Levels

When the experiment was terminated at the end of the 13^th^ week, serum was collected from each group (2000 rpm, 15 min, 4°C). Levels of CRP, IL-6, TNF-*α*, MDA, and SOD in serum were analyzed with appropriate ELISA kits based on provided directions.

### 2.6. Quantitative PCR

Rat aorta (80 mg) of the CON, MOD, and AVF groups was used for RNA extraction using 1 ml TRIzol (Invitrogen, USA). mRNA expression was quantified using the TransScript Green Two-Step qRT-PCR Supermix (TransGen Biotech, Beijing, China). All primers were obtained from GeneCopoeia (USA). The sequences of primers are listed as follows: the ICAM-1 primer sequences were as follows: forward primer 5′-CGTGACCTGGACACACCTAC-3′ and reverse primer 5′-TGTCCCAGCTTTCCCATCTC-3′. The VCAM-1 primer sequences were as follows: forward primer 5′-CTACATGAGGGTGCTGCTGT-3′ and reverse primer 5′-GAACAACGGAATCCCCAACC-3′. The E-selectin primer sequences were as follows: forward primer 5′-CCACATGTGCAGGGGTACAG-3′ and reverse primer 5′-ATCCGTTGAGTGTCCAACCC-3′. GAPDH was used as an internal reference; the primer sequences were as follows: forward primer 5′-GTTACCAGGGCTGCCTTCTC-3′ and reverse primer 5′-GATGGTGATGGGTTTCCCGT-3′. The PCR conditions were as follows: denaturation at 94°C for 30 s, followed by 45 cycles at 94°C for 5 s, 60°C for 15 s, and 72°C for 10 s; the CT value of each sample was recorded. Based on the CT values for the target gene and reference genes, we used 2^−ΔΔ*CT*^ to represent the relative expression levels of the target gene, according to ΔΔCT = (CT target − CT reference) experiment − (CT target − CT reference) control.

### 2.7. Western Blot Analysis

A rat aortic sample (100 mg) was diced, placed in 1 ml of RIPA lysis buffer (containing one *μ*mol/L PMSF), and fully homogenized, followed by centrifugation at 12,000 g for 20 min. A total of 100 *μ*g of total protein per sample was separated on 10% sodium dodecyl sulfate-polyacrylamide gels by electrophoresis at 120 V for one hour, followed by a transfer onto polyvinylidene difluoride membranes at 100 V for one hour. The membranes were then blocked with 5% nonfat dry milk in Tris-buffered saline containing Tween 20 (0.15 M NaCl, 20 mM Tris-HCl, pH 7.4, and 0.05% Tween 20) for one hour at room temperature, followed by incubation with specific primary antibodies (anti-p38, anti-FKN, and anti-SYK; 1 : 1000 dilution; Abcam, USA) at 4°C overnight. Then, the membranes were incubated with a horseradish peroxidase-conjugated secondary antibody (1 : 5000 dilution; Santa Cruz Biotechnology, USA). The specific protein bands were detected with enhanced chemiluminescence reagent (Amersham, USA). GAPDH antibody (Sigma, USA) was used as an internal control.

### 2.8. Statistical Analysis

All statistical analyses were carried out using the statistical package SPSS 19.0 (IBM Corp., USA). Data were presented as the mean ± standard deviation (SD) (*n* = 12). Multiple groups were compared using the one-way analysis of variance followed by the least significant difference test. Statistical significance was defined as *p* < 0.05.

## 3. Results

### 3.1. Comparison of the General Condition and Blood Lipid Levels of the Rats

As shown in Figure 1(a), the rats showed slow weight gain after feeding with high-fat diets. Starting from the 3^rd^ week, the weight of rats on the high-fat diet was significantly lower than that of the CON group (*p* < 0.01) fed with the usual diet, and there was no significant difference in the body weight of the other groups.

In this experiment, the ELISA method was used to detect blood lipids in the serum of rats. As shown in Figure 1(b), when the experiment ended in the 13^th^ week, the serum TC, TG, LDL-C, and HDL-C levels of each group of rats were detected. It was found that compared with the CON group, the serum TG, TC, and LDL-C contents of the MOD group were significantly increased, while the HDL-C level was significantly decreased (*p* < 0.01). Compared with the MOD group, serum TG, TC, and LDL-C levels in the SIM group and each dose group of AVF were reduced to different degrees, and the level of HDL-C increased.

### 3.2. Histological Examination of the Rats' Aorta Tissue

HE staining can show the extent of organ lesions. In this study, the HE method was used to observe the aorta. As Figure 2 shows, the tunica intimae of aortas in the normal group were smooth without lipid deposition and contained a small number of collagen fibers and soft muscle fibers, as well as uniformly distributed elastic fibers. The rats in the untreated atherosclerosis group showed obvious atherosclerosis. Those with mild symptoms showed increased lipids and various numbers of visible foam cells. Those with severe symptoms presented arterial wall calcification. Rats in the *Apocynum* and the simvastatin groups also showed various degrees of atherosclerotic lesions in the arterial wall; the calcification lesions were significantly lower, and the extent of calcification was considerably less than that of those in the untreated atherosclerosis group.

### 3.3. Serum Inflammatory Factors, SOD, and MDA Levels

In this experiment, ELISA was used to detect oxidative stress and inflammation-related indicators in rat serum. As shown in Figure 3, compared with the CON group, the content of CRP, IL-6, TNF-*α*, and MDA in the MOD group was significantly increased (*p* < 0.001), and the SOD level was reduced significantly (*p* < 0.001); compared with the MOD group, the SIM group and medium-AVF and high-AVF groups can significantly reduce the levels of CRP, IL-6, TNF-*α*, and MDA (*p* < 0.001) and increase the content of SOD (*p* < 0.001). At the same time, the above indicators of low AVF have not changed significantly.

### 3.4. Expression of ICAM-1, VCAM-1, and E-Selectin mRNA and Protein in the Rat Thoracic Aorta

Real-time PCR and western blot were used to detect the expression levels of ICAM-1, VCAM-1, and E-selectin mRNA and protein in the thoracic aorta of each group. The results (Figure 4) found that compared with the CON group, the expression levels of ICAM-1, VCAM-1, and E-selectin in the thoracic aorta of the MOD group were significantly increased (*p* < 0.001); compared with the MOD group, the expression levels of ICAM-1, VCAM-1, and E-selectin in the thoracic aorta of the medium-AVF and high-AVF groups were decreased significantly (*p* < 0.001). In contrast, the indicators of the low-AVF group had no significant improvement (*p* > 0.05).

### 3.5. Effects of FKN, SYK, and p38MARK Protein Expression

Western blotting was used to detect the expression of FKN, p-SYK, and p-p38 protein in the thoracic aorta of each group. The results (Figure 5) showed that compared with the CON group, the expression of FKN, p-SYK, and p-p38 protein levels in the thoracic aorta increased in the MOD group (*p* < 0.001); compared with the MOD group, the expression of FKN, p-SYK, and p-p38 protein levels in the thoracic aorta of the low-AVF, medium-AVF, and high-AVF groups and SIM group was significantly decreased (*p* < 0.01); and the expression of three proteins in medium-AVF and high-AVF groups was lower than that in the low-AVF group.

## 4. Discussion

Atherosclerosis is a chronic multifactorial disease that has high morbidity and mortality. It is well known that elevated serum cholesterol levels and proinflammatory factors drive atherogenesis [4]. Flavonoids, a common component of many Chinese traditional herbs, have been shown to interfere with the progression of AS [15], as evidenced by the findings that flavonoids can reduce vascular fragility and abnormal permeability [5, 6, 8, 16], but the effects of total flavonoids from the *Apocynum venetum* leaf on the pathogenesis of AS and the underlying mechanisms have not been well studied. In our study, we found that AVF treatment significantly ameliorated hyperlipidemia, inflammation, and adhesion factors in a rat AS model induced by an HCD and VD_3_, suggesting that AVF can attenuate the initiation and progression of AS.

Disturbance of lipid metabolism is directly related to the development of AS [17–19]. In the early stages of AS, abnormal lipid metabolism can damage vascular endothelial cells (VECs) and cause dysfunction, which in turn causes the expression of inflammatory factors and adhesion molecules and, at the same time, promotes the proliferation and migration of vascular smooth muscle cells (VSMCs) and the formation of foam cell AS [20]. After feeding with high-fat diets, the rats showed slow weight gain. Starting from the 3^rd^ week, the weight of rats on the high-fat diet was significantly lower than that of the CON group (*p* < 0.01) fed with the usual diet, and there was no significant difference in the body weight of the other groups. This result may be because the high-fat feed completely replaced the ordinary meal, and the addition of cholate and propylthiouracil made the rat unsuitable for its taste. The reduction in food intake led to a significant decrease in the weight of the high-fat diet rats. In addition, when lipid metabolism is increased, LDL can be oxidatively modified to form Ox-LDL, which can induce dysfunction of VECs and migration and proliferation of VSMCs. Therefore, the disorder of lipid metabolism plays a vital role in the development of AS. In this study, different AVF doses were used to intervene in AS rats. After four weeks of AVF treatment, the levels of TC, TG, and LDL in AS rats were significantly reduced, while HDL levels were significantly increased. Pathological observation of the rat thoracic aorta showed that AVF could significantly reduce the pathological damage of the thoracic aorta of AS rats, inhibit inflammatory cell infiltration, reduce foam-like cell generation, inhibit smooth muscle cell proliferation, and reduce atrophy of the media. The above results indicate that AVF can treat AS model rats by lowering blood lipid levels.

Oxidative stress is closely related to AS [21]. Excessive ROS can promote the production of Ox-LDL, and Ox-LDL is an essential initiating factor of AS inflammation. SOD is an essential antioxidant enzyme in the body, removing excessive ROS in cells [4]. MDA is the final product of the peroxidation of polyvalent unsaturated fatty acids initiated by free radicals in the body. Both SOD and MDA can directly or indirectly reflect the effects of drugs on lipid peroxidation. Under normal physiological conditions, the body maintains a dynamic balance between oxidation and antioxidation. Once the balance is destroyed, oxidative stress will produce excessive ROS and active nitrogen, resulting in the formation of many free radicals and nonfree radicals, damaging cells [22, 23]. Some studies have shown that, in AS animal models, as the blood lipid level of rabbits increases, SOD activity decreases, and MDA content increases [24]. In this study, the serum SOD activity and MDA content of rats were detected. The results showed that the MOD group had significantly reduced serum SOD activity and significantly increased MDA levels. After AVF intervention, it can significantly increase SOD activity and reduce MDA content, suggesting that AVF can achieve an anti-AS effect by inhibiting oxidative stress response.

The inflammatory response involves every stage of AS occurrence. The inflammatory factors CRP, IL-6, and TNF-*α* play a vital role in the occurrence and development of AS diseases and are closely related to the formation of AS. CRP is directly involved in all critical stages of AS pathogenesis, and it is a susceptible detection index in the occurrence and development of AS [25]. CRP can increase the expression of ROS and Ox-LDL and aggravate vascular inflammation [26]. IL-6 is a pleiotropic proinflammatory cytokine. In the process of AS, TNF-*α* can increase leukocyte chemotaxis by inducing platelet adhesion, promote the adhesion of monocytes to endothelial cells, promote blood coagulation, and participate in the occurrence of AS [27]. This study found that the serum CRP, IL-6, and TNF-*α* expressions of AS rats were significantly increased, suggesting an inflammatory response in the thoracic aorta of AS rats. However, AVF can substantially reduce CRP, IL-6, and TNF-*α*, suggesting that AVF can reduce the expression of serum CRP, IL-6, and TNF-*α* to reduce the inflammation and then achieve the anti-AS effect.

ICAM-I and VCAM-1 promote the adhesion of monocytes on the surface of VECs, enter the endothelium and transform into macrophages, engulf Ox-LDL to form foam cells, and, at the same time, promote platelet adhesion, activation, and thrombosis, producing a variety of growth factors that promote the proliferation of VSMCs in AS plaques [28]. E-selectin belongs to the selectin superfamily of adhesion molecules, and its function is to promote the adhesion of leukocytes to VECs [29]. In this study, real-time PCR technology was used to detect the gene expression of ICAM-1, VCAM-1, and E-selectin in rat thoracic aorta tissue. The gene expression of ICAM-1, VCAM-1, and E-selectin decreased significantly, suggesting that AVF can control the development of AS by inhibiting the expression of adhesion molecules, reducing the adhesion between VECs and leukocytes, and inhibiting the inflammatory response.

AS is a chronic inflammatory disease, not only caused by the simple deposition of lipids on the blood vessel wall. There are multiple signaling pathways involved in the evolution of inflammation. FKN is a chemokine with both adhesion and chemotactic activity and plays an important role in the migration of vascular smooth muscle cells to atherosclerotic plaques [30]. SYK is a nonreceptor tyrosine kinase, expressed in a variety of cells, mainly related to the inflammatory process. SYK plays a critical regulatory role in the inflammatory process of atherosclerosis, such as oxidized lipid deposition, C-reactive protein, NF-*κ*B activation, platelet activation, and inflammatory body activation [31, 32]. In every stage of AS, p38 can promote the secretion of chemokines and inflammatory mediators and encourage the adhesion of monocytes and the formation of foam cells [33–36]. FKN released by endothelial cells can bind to its receptor CX3CR1, resulting in endothelial cell damage. It can make monocytes and lymphocytes expressing CX3CR1 chemotaxis adhere to and migrate toward vascular endothelial cells, thereby initiating atherosclerosis [37]. And FKN can mediate SYK to induce the expression of p38 and participate in the occurrence and development of AS through inflammatory mechanisms. Studies have confirmed that SYK is one of the upstream signal molecules of the p38 signal transduction pathway. It is clear that FKN stimulates mononuclear cells to cause p38 activation. The FKN/SYK/p38 signaling pathway is related to the occurrence and development of AS, that is, FKN can induce the expression of p38 through Syk and induce the expression of related inflammatory factors through Syk and p38 to induce AS [38, 39]. In this experiment, western blotting was used to detect the expression of FKN, p-SYK, and p-p38 proteins in the rat thoracic aorta. The results showed that the AVF in each treatment group could reduce the expression levels of FKN, p-SYK, and p-p38 proteins, and the effect was similar to that of the positive drug simvastatin, suggesting that the AVF could be the anti-FKN/SYK/p38 signaling pathway.

In summary, AVF mainly exerts its anti-AS effects by reducing blood lipids and MDA levels, increasing SOD levels, and reducing serum inflammatory factors CPR, IL-6, and TNF-*α* and cell adhesion molecules ICAM-1, VCAM-1, and E-selectin effect. At the same time, the experiment found that AVF can play an anti-AS role by inhibiting the FKN/SYK/p38 signaling pathway.

## Figures and Tables

**Figure 1:** Comparison of the body weight and the blood lipid of the rats in various groups. (a) Body weight of rats. (b) Rats' blood lipids. CON: control group; MOD: model group; SIM: simvastatin group; low AVF, medium AVF, and high AVF: *Apocynum* leaf flavonoids' low-, medium-, and high-dose treated group. ^*∗*^*p* < 0.05, ^*∗∗*^*p* < 0.01, and ^*∗∗∗*^*p* < 0.001 as compared with the CON group; ^#^*p* < 0.05, ^##^*p* < 0.01, and ^###^*p* < 0.001 as compared with the MOD group; ^△^*p* < 0.05, ^△△^*p* < 0.01, and ^△△△^*p* < 0.001 as compared with the SIM group.

**Figure 2:** Hematoxylin-eosin (HE) staining results in the rats of various groups (×200). CON: control group; MOD: model group; SIM: simvastatin group; low AVF, medium AVF, and high AVF: *Apocynum* leaf flavonoids' low-, medium-, and high-dose treated group. (a) CON, (b) MOD, (c) SIM, (d) low AVF, (e) medium AVF, and (f) high AVF.

**Figure 3:** Levels of inflammatory factors and oxidative stress in serum of rats in each group. (a) Serum CRP levels; (b) serum IL-6 levels; (c) serum TNF-*α* levels; (d) serum SOD levels; (e) serum MDA levels. CON: control group; MOD: model group; SIM: simvastatin group; low AVF, medium AVF, and high AVF: *Apocynum* leaf flavonoids' low-, medium-, and high-dose treated group. ^*∗*^*p* < 0.05, ^*∗∗*^*p* < 0.01, and ^*∗∗∗*^*p* < 0.001 as compared with the CON group; ^#^*p* < 0.05, ^##^*p* < 0.01, and ^###^*p* < 0.001 as compared with the MOD group; ^△^*p* < 0.05, ^△△^*p* < 0.01, and ^△△△^*p* < 0.001 as compared with the SIM group.

**Figure 4:** Real-time and western blot results of ICAM-1, VCAM-1, and E-selectin in the aortic wall. (a) ICAM-1 mRNA expression; (b) VCAM-1 mRNA expression; (c) E-selectin mRNA expression; (d) ICAM-1 protein expression; (e) VCAM-1 protein expression; (f) E-selectin protein expression. CON: control group; MOD: model group; SIM: simvastatin group; low AVF, medium AVF, and high AVF: *Apocynum* leaf flavonoids' low-, medium-, and high-dose treated group. ^*∗*^*p* < 0.05, ^*∗∗*^*p* < 0.01, and ^*∗∗∗*^*p* < 0.001 as compared with the CON group; ^#^*p* < 0.05, ^##^*p* < 0.01, and ^###^*p* < 0.001 as compared with the MOD group; ^△^*p* < 0.05, ^△△^*p* < 0.01, and ^△△△^*p* < 0.001 as compared with the SIM group.

**Figure 5:** Western blot results of FKN, p-SYK, and p-p38 in the aortic wall. (a) Representative FKN and GAPDH ratio. (b) Representative SYK and p-SYK ratio. (c) Representative p38 and p-p38 ratio. CON: control group; MOD: model group; SIM: simvastatin group; low AVF, medium AVF, and high AVF: *Apocynum* leaf flavonoids' low-, medium-, and high-dose treated group. ^*∗*^*p* < 0.05, ^*∗∗*^*p* < 0.01, and ^*∗∗∗*^*p* < 0.001 as compared with the CON group; ^#^*p* < 0.05, ^##^*p* < 0.01, and ^###^*p* < 0.001 as compared with the MOD group; ^△^*p* < 0.05, ^△△^*p* < 0.01, and ^△△△^*p* < 0.001 as compared with the SIM group.

## Data Availability

The datasets used and/or analyzed during the present study are available from the corresponding author upon reasonable request.
